# Assessment of the SFlt-1 and sFlt-1/25(OH)D Ratio as a Diagnostic Tool in Gestational Hypertension (GH), Preeclampsia (PE), and Gestational Diabetes Mellitus (GDM)

**DOI:** 10.1155/2019/5870239

**Published:** 2019-08-06

**Authors:** Malgorzata Walentowicz-Sadlecka, Piotr Domaracki, Pawel Sadlecki, Joanna Siodmiak, Marek Grabiec, Pawel Walentowicz, Maria Teresa Arias Moliz, Grazyna Odrowaz-Sypniewska

**Affiliations:** ^1^Department of Obstetrics and Gynecology, L. Rydygier Collegium Medicum in Bydgoszcz, Nicolaus Copernicus University, ul. Ujejskiego 75, Bydgoszcz 85-168, Poland; ^2^Department of Laboratory Medicine, L. Rydygier Collegium Medicum in Bydgoszcz, Nicolaus Copernicus University, M. Curie Skłodowskiej 9, Bydgoszcz 85-094, Poland; ^3^Department of Microbiology, University of Granada, Avda. del Hospicio, 18071 Granada, Spain

## Abstract

**Background:**

Placental soluble fms-like tyrosine kinase-1 (sFlt-1), an antagonist of vascular endothelial growth factor, is considered an etiological factor of endothelial damage in pregnancy pathologies. An increase in the sFlt-1 level is associated with alterations of endothelial integrity. In contrast, vitamin D exerts a protective effect and low concentrations of 25(OH)D may have an adverse effect on common complications of pregnancy, such as gestational hypertension (GH), preeclampsia (PE), and gestational diabetes mellitus (GDM). The aim of this study was to analyze the levels of sFlt-1 in Polish women with physiological pregnancies and pregnancies complicated by GH, PE, and GDM. Moreover, we analyzed relationships between the maternal serum sFlt-1 level and the sFlt-1 to 25(OH)D ratio and the risk of GH and PE.

**Material and Methods:**

The study included 171 women with complicated pregnancies; among them are 45 with GH, 23 with PE, and 103 with GDM. The control group was comprised of 36 women with physiological pregnancies. Concentrations of sFl-1 and 25(OH)D were measured before delivery, with commercially available immunoassays.

**Results:**

Women with GH differed significantly from the controls in terms of their serum sFlt-1 levels (5797 pg/ml vs. 3531 pg/ml, *p* = 0.0014). Moreover, a significant difference in sFlt-1 concentrations was found between women with PE and those with physiological pregnancies (6074 pg/ml vs. 3531 pg/ml, *p* < 0.0001). GDM did not exert a statistically significant effect on serum sFlt-1 levels. Both logistic regression and ROC analysis demonstrated that elevated concentration of sFlt-1 was associated with greater risk of GH (AUC = 0.70, *p* = 0.0001) and PE (AUC = 0.82, *p* < 0.0001). Also, the sFlt-1 to 25(OH)D ratio, with the cutoff values of 652 (AUC = 0.74, *p* < 0.0001) and 653 (AUC = 0.88, *p* < 0.0001), respectively, was identified as a significant predictor of GH and PE.

**Conclusions:**

Determination of the sFlt-1/25(OH)D ratio might provide additional important information and, thus, be helpful in the identification of patients with PE and GH, facilitating their qualification for intensive treatment and improving the neonatal outcomes.

## 1. Introduction

Preeclampsia (PE) and gestational diabetes mellitus (GDM) are two of the most important causes of pregnancy complications. The incidence of both these conditions has been gradually increasing worldwide, up to 5% for PE and up to 13% for GDM [1, 2]. Gestational hypertension (GH) is a leading cause of morbidity and mortality in pregnant women, fetuses, and newborns [3]. PE manifests after 20 weeks of gestation and constitutes a life-threatening condition for both fetuses and pregnant women. The prevalence of GH increases with age and is higher in overweight and obese women [4].

The term “diabetes” refers to a group of metabolic diseases associated with hyperglycemia resulting from impaired secretion or function of insulin [5]. To be classified as gestational, diabetes needs to be detected for the first time during pregnancy [6]; the proportion of pregnancies complicated by GDM is estimated at 3-12% [7]. Aside from patient's age, the risk of GDM increases with body weight and is particularly high in obese women. A British population-based study demonstrated that the proportion of obese pregnant women has nearly doubled, from 9-10% in early 1990's to 16-19% in the first years of the 21^st^ century [8]. Pregnant women with GDM are at increased risk of GH and PE; insulin resistance and hyperglycemia are associated with greater oxidative stress which contributes to endothelial dysfunction in blood vessels and predisposes to hypertension [9].

An antiangiogenic factor, soluble fms-like tyrosine kinase 1 (sFlt-1), was shown to play an important role in the pathogenesis of many conditions related to vascular endothelium. sFlt-1 is an endogenous inhibitor of vascular endothelial growth factor (VEGF). Binding to VEGF proteins, sFlt-1 reduces their pool that can interact with transmembrane receptors and, hence, attenuates the VEGF-mediated signaling [10]. This contributes to impairment of angiogenesis and greater vascular permeability leading to the loss of serum proteins [11]. Available evidence suggests that elevated levels of sFlt-1 might be associated with the occurrence of PE and other pregnancy complications, such as intrauterine growth restriction, preterm labor, and miscarriage [12]. Importantly, an increase in the sFlt-1 level can be observed well before the first clinical manifestations of gestational complications, which implies that this parameter could be used to distinguish between physiological and high-risk pregnancies [13].

Vitamin D deficiency is associated with endothelial dysfunction. Epidemiological studies demonstrated a link between the low maternal level of vitamin D and higher incidence of GH and showed that deficiency of this vitamin may be an independent risk factor of PE [14]. Activation of vitamin D receptors is known to promote VEGF expression; further, an adequate level of vitamin D and appropriate expression of vitamin D receptors (VDRs) were shown to be fundamental for angiogenic function of endothelial cells and their protection against oxidative damage [15]. In our previous study, we found a significant association between the low serum level of vitamin D and the risk of preeclampsia; the area under ROC curve (AUC) for serum vitamin D as a predictor of PE was 70.3% [16].

The aim of this study was to analyze serum levels of sFlt-1 and the values of the sFlt-1 to 25(OH)D ratio in Polish women with physiological pregnancies and pregnancies complicated by GH, PE, and GDM. Identification of a link between the sFlt-1 level and the risk of pregnancy complications could play an important role in the prediction of their occurrence, thus, contributing to better outcomes in pregnant women and their offspring.

## 2. Materials and Methods

The study, conducted in 2013-2015 at the Department of Obstetrics and Gynecology, Ludwik Rydygier Collegium Medicum in Bydgoszcz, Nicolaus Copernicus University of Torun, included 207 women with singleton pregnancies (all Caucasians of Polish nationality, residents of Kuyavian-Pomeranian Province). The age of the study participants ranged between 19 and 40 years.

The study group included 171 women—45 patients with GH, 23 with PE, and 103 with GDM. Women who presented with concomitant GH and GDM were excluded from the study. GH was defined as a systolic blood pressure > 140 mmHg or diastolic blood pressure > 90 mmHg on two or more measurements at least six hours apart, occurring after 20 weeks of gestation, without concomitant proteinuria. PE was defined as the onset of hypertension (systolic blood pressure ≥ 140 mmHg or diastolic blood pressure ≥ 90 mmHg) in a previously normotensive woman, coexisting with proteinuria (at least 0.3 g of protein in a 24-hour urine sample) without a concomitant urinary tract infection. GDM was detected based on the result of a 75 g oral glucose tolerance test (OGTT) conducted between 24 and 28 weeks of gestation. Women with GDM were stratified according to the type of this condition, G1 or G2, in line with the White classification [6]. Type A1 (corresponding to GDM G1) was defined as an abnormal result of OGTT, normal blood glucose levels during fasting and one/two hours after a meal, and the ability to control glycemia solely with a dietary modification. Type A2 (corresponding to GDM G2) was defined as an abnormal result of OGTT, abnormal glucose levels during fasting and/or after a meal, and the inability to control glycemia without additional therapy with insulin or other agents. All study patients presented with appropriate-for-gestational-age (AGA) pregnancies. Women after in vitro fertilization, as well as those with comorbidities, were excluded from the study. Serum concentrations of sFlt-1 and 25(OH)D were determined during hospital stay shortly before delivery. Women who presented with abnormal blood pressure were additionally examined for the severity of GH and the presence of PE. Other clinicodemographic variables included in the analysis were maternal age, parity, body mass index (BMI), gestational age at delivery, route of delivery, birth weight, and pH of the umbilical cord blood. The control group included 36 women with uncomplicated pregnancies, normal arterial blood pressure, and glucose concentrations. All blood samples were obtained in the third trimester, 1-7 days before delivery. All controls were matched for the gestational age.

### 2.1. Methods

10 ml blood samples were obtained from the cubital vein and immediately separated by centrifugation. The sera were stored at -80°C until the analysis. Serum concentrations of sFlt-1 were determined with the fully automated Elecsys® electrochemiluminescence assay (Roche Diagnostics, Manheim, Germany). The assay was performed using Roche immunoanalyzer Elecsys® 2010/cobas e411, in line with the manufacturer's instruction. The detection range of the assay was 10-85 000 pg/ml, and the limit of quantification amounted to 15 pg/ml. Interassay coefficient of variation (CV) for the sFlt-1 assay was 4.3% at a mean concentration of 98 pg/ml (PreciControl Multimarker 1, Roche Diagnostics, Manheim, Germany) and 3.8% at 1 020 pg/ml (PreciControl Multimarker 2, Roche Diagnostics, Manheim, Germany). The limit of detection for the test was 10 pg/ml. Serum 25(OH)D concentration was determined by ELISA (25-hydroxy vitamin D EIA), Immunodiagnostic Systems Ltd., in the Department of Laboratory Diagnostics, Ludwik Rydygier Collegium Medicum, Nicolaus Copernicus University in Torun; the sensitivity was 2.0 ng/ml (5 nmol/l) and the assay measured range was 2.7–152 ng/ml (6.8–380 nmol/l). A certified reference material (NIST Standard Reference Material (SRM) 972) was used for vitamin D measurement. The method remained under RIQAS control, and the results of the assay are within the reference range for this control. The inter- and intraassay variabilities were 5.3% and 4.6%. A concentration of 25(OH)D < 10 ng/ml (<25 nmol/l) was defined as deficiency, 10–29 ng/ml (25–74 nmol/l) has been accepted as insufficiency, and sufficient was when concentrations were between 30 and 100 ng/ml (75–250 nmol/l). In our previous study, we presented levels of serum vitamin D levels in all study subgroups [16].

### 2.2. Statistical Analyses

Statistical analyses were carried out with PQStat software, version 1.6. The significance of intergroup differences in sFlt-1 concentrations was verified with Mann-Whitney *U* test and Kruskal-Wallis test with Dunn's post hoc tests. Direction and power of relationships between serum sFlt-1, maternal age, pH of the umbilical cord blood, and birth weight were estimated based on Spearman's coefficients of rank correlation. Statistical significance of potential predictors of GH, PE, and GDM were verified in univariate and multivariate models of logistic regression. The roles of sFlt-1 and the sFlt-1 to 25(OH)D ratio as predictors of GH and PE were additionally verified on ROC analysis. The results of all the tests were considered significant at *p* < 0.05 and highly significant at *p* < 0.01.

The protocol of the study was approved by the Local Bioethics Committee at Ludwik Rydygier Collegium Medicum in Bydgoszcz (decision no. KB 502/2013), and written informed consent was sought from all participants.

## 3. Results

Patient age, parity, BMI, gestational age at delivery, route of delivery, birth weight, and pH of the umbilical cord blood were analyzed. The control group included 36 women with uncomplicated pregnancies, normal arterial blood pressure, and glucose concentrations. Baseline characteristics of study participants are presented in Table 1.

Women with GH differed significantly from the controls in terms of their sFlt-1 concentrations (5797 pg/ml vs. 3531 pg/ml, *p* = 0.0014; Table 2). Similarly, a significant difference was found between sFlt-1 concentrations in women with PE and the controls (6074 pg/ml vs. 3531 pg/ml, *p* < 0.0001; Table 3). However, no statistically significant differences were observed between sFlt-1 concentrations in women with GDM G1, women with GDM G2 and the controls (4301 pg/ml vs. 3704 pg/ml vs. 3531 pg/ml, *p* = 1.0000; Table 4).

While we must admit that our control group was relatively small (*N* = 36), the results for this group are consistent with those reported by other authors and fit within published reference limits for the third trimester [17].

Table 5 presents sFlt-1 concentrations stratified according to arterial pressure of the study participants. The levels of sFlt-1 increased with blood pressure and were the highest in the group of patients whose blood pressure exceeded 180/110 mmHg.

We also compared sFlt-1 levels in the groups of patients with adequate serum concentrations of 25(OH)D (≥20 ng/mL) and vitamin D deficiency. The results are presented in Table 6. The concentrations of sFlt-1 in patients with adequate serum levels of 25(OH)D (≥20 ng/ml) turned out to be significantly lower than in those with vitamin D insufficiency/deficiency (3356 pg/ml vs. 4452 pg/ml, *p* = 0.0256).

Then, we conducted a series of ROC analyses to verify whether sFlt-1 and the sFlt-1 to 25(OH)D ratio were significant predictors of GH and PE. The results are presented in Tables 7 and 8. Serum sFlt-1 turned out to be a significant predictor of GH (*p* = 0.001) and PE (*p* < 0.0001), with AUC equal 70.1% and 82.4, respectively (Figures 1 and 2). Also, the sFlt-1 to 25(OH)D ratio was identified as a significant predictor of both GH (*p* < 0.0001) and PE (*p* < 0.0001), with AUC amounting to 73.6% and 87.96%, respectively (Figures 3 and 4). In our present study, the serum sFlt-1 to 25(OH)D ratio (with the cutoff value of 652) was identified as a good predictor of GH on ROC analysis (*p* < 0.0001), with an AUC equal 73.6%. Moreover, the serum sFlt-1 to 25(OH)D ratio (with a similar cutoff value as above, 653) turned out to be a significant predictor of PE (*p* < 0.0001), with an AUC equal 87.96%.

Finally, multivariate logistic regression analysis was conducted to verify if serum sFlt-1 predicted GH and PE independently from other established risk factors (BMI ≥ 30 kg/m^2^, age ≥ 35 years, primiparity) and low vitamin D levels. The results are presented in Tables 9 and 10. On multivariate logistic regression analysis, 25(OH)D was not identified as an independent predictor of either hypertension or preeclampsia (*p* > 0.05). The analysis identified serum sFlt-1 and BMI ≥ 30 kg/m^2^ as independent predictors of GH. Furthermore, serum sFlt-1 turned out to be an independent predictor of PE on multivariate logistic regression analysis.

## 4. Discussion

Impaired synthesis of placental biomarkers and vitamin D deficiency have been postulated as risk factors of many pregnancy pathologies; however, in the case of many such relationships, the exact pathogenic mechanisms are not fully understood. A growing body of evidence suggests that endothelial dysfunction may play an important role in the pathogenesis of many pregnancy complications [18].

VEGFs are essential for proper implantation of the placenta. Soluble type 1 receptor for VEGF (soluble fms-like tyrosine kinase 1 (sFlt-1)) probably plays an important role in many processes occurring during pregnancy, modulating function of VEGFs [19]. Placental ischemia was shown to be associated with the production of factors contributing to endothelial dysfunction, among them sFlt-1; the dysfunction of vascular endothelium can manifest as arterial hypertension and proteinuria [20–22].

Considering the results of many previous studies that documented the link between the sFlt-1 status and the occurrence of pregnancy pathologies, we verified whether a similar relationship existed in Polish women with GH. Our study showed that sFlt-1 concentrations in women with GH were significantly higher than in those with physiological pregnancies (5797 pg/ml vs. 3531 pg/ml, *p* = 0.0014) and serum sFlt-1 was identified as a significant predictor of GH on both logistic regression analysis and ROC analysis. On ROC analysis, serum sFlt-1 turned out to be a significant predictor of GH (*p* = 0.001), with an AUC equal 70.1%. Furthermore, multivariate logistic regression analysis identified elevated serum sFlt-1 and BMI ≥ 30 kg/m^2^ as independent predictors of GH.

Our findings are consistent with the results published by Nanjo et al. [23] who demonstrated that prior to delivery, women with GH presented with significantly higher sFlt-1 levels than those without. Moreover, they found a significant correlation between the levels of circulating angiogenic factors shortly before delivery and the severity of hypertensive disorders in pregnancy [23]. Also, in our study, sFlt-1 concentrations increased with maternal blood pressure and were the highest in patients with arterial pressure exceeding 180/110 mmHg. This might be another argument for a role of sFlt-1 in endothelial damage. Possibly, the higher the blood pressure, the greater the endothelial damage and the more elevated the sFlt-1 levels. Our findings are consistent with the results of many previously published studies [24]. According to Verlohren et al., the sFlt-1/PlGF ratio allowed the identification of women at risk for imminent delivery and was a reliable tool to discriminate between various types of pregnancy-related hypertensive disorders [24].

Both available evidence and our present findings imply that sFlt-1 plays an important role in the pathogenesis of GH and PE, as well as in the clinical course of these conditions [25]. PE is diagnosed whenever a pregnant woman presents with hypertension and concomitant proteinuria. The proteinuria may be a consequence of glomerular damage which can be caused by binding sFlt-1 to VEGF and resultant destruction of vascular endothelium. The same mechanism may also be involved in glomerular damage in patients with GDM [26].

In this context, it is not surprising that patients with PE presented with the highest sFlt-1 concentrations of all pregnant women participating in our study. The concentration of sFlt-1 in the PE group turned out to be significantly higher than in the controls (6074 pg/ml vs. 3531 pg/ml, *p* < 0.0001). Furthermore, serum sFlt-1 was identified as a significant determinant of PE on ROC analysis (*p* < 0.0001), with AUC equal 82.4%. Serum sFlt-1 was also identified as an independent predictor of PE on multivariate logistic regression analysis. The elevated serum level of sFlt-1 was shown to be associated with higher risk of PE. sFlt-1 is known to contribute to endothelial damage, and hence, an increase in its concentration may negatively affect vascular integrity. The role of sFlt-1 in PE was a subject of many previous studies. Agrawal et al. conducted a meta-analysis to explore the predictive value of the sFlt-1/PlGF ratio in preeclampsia. The meta-analysis included 15 studies with a total of 534 cases of preeclampsia and 19587 controls. The sFlt-1/PlGF ratio had a pooled sensitivity of 80% (95% confidence interval, 0.68-0.88), specificity of 92% (95% confidence interval, 0.87-0.96), positive likelihood ratio of 10.5 (95% confidence interval, 6.2-18.0), and a negative likelihood ratio of 0.22 (95% confidence interval, 0.13-0.35) in predicting preeclampsia in both high- and low-risk patients. According to the authors of the meta-analysis, these findings imply that the sFlt-1/PlGF is a valuable screening tool for preeclampsia and might be helpful in decision-making, treatment stratification, and better resource allocation [27].

A recent prospective multicenter observational study PROGNOSIS (prediction of short-term outcome in pregnant women with suspected preeclampsia study) was designed to analyze the serum sFlt-1 to placental growth factor (PlGF) ratio as a predictor of PE during a short-term follow-up of women with singleton pregnancies (24 weeks and 0 days to 36 weeks and 6 days of gestation) suspected of this condition [28]. The study demonstrated that the sFlt-1 to PlGF ratio of 38 or less might be used to exclude PE in a short-term perspective in women suspected of this condition based on clinical presentation.

Although the role of the sFlt-1 to PlGF ratio raises no controversies, we still need more data about other potential predictors of GH and PE. Specifically, a reliable predictor of PE (and in particular the absence thereof) is needed in women with clinical suspicion of this pregnancy complication. Many women whose clinical presentation raises a suspicion of PE are hospitalized until this condition and other adverse outcomes have been excluded. At the same time, PE may be overlooked in other pregnant women who should be hospitalized. Although no preventive or therapeutic strategy for PE is yet available except low-dose acetylsalicylic acid treatment which was shown to exert a moderate preventive effect on high-risk pregnancies after the first trimester, clinical experience suggests that early detection and monitoring could be beneficial. Therefore, based on published evidence including the results of our previous study [16], we decided to verify whether sFlt-1 and 25(OH)D concentrations might be used as the measures of GH and pH risk. Our study demonstrated that women with adequate serum levels of 25(OH)D (≥20 ng/ml) presented with significantly lower levels of sFlt-1 than those with vitamin D deficiency (3356 pg/ml vs. 4452 pg/ml, *p* = 0.0256). This observation is consistent with the results published by Zeisler et al. [28]. According to those authors, 25(OH)D concentrations in women diagnosed with PE were significantly lower than those in patients without this condition and a low level of 25(OH)D was associated with increased risk of late-onset PE (odds ratio 4.6, 95% confidence interval 1.4-15). Interestingly, however, no similar association was found for early-onset PE. Furthermore, the study did not demonstrate a link between the 25(OH)D level and the sFlt-1 to PlGF ratio. Based on those findings, Álvarez-Fernández et al. concluded that low concentration of vitamin D in women with suspected late-onset PE is associated with increased risk of the imminent disease [29].

In our present study, the serum sFlt-1 to 25(OH)D ratio (with the cutoff value of 652) was identified as a good predictor of GH on ROC analysis (*p* < 0.0001), with an AUC equal 73.6%. Moreover, the serum sFlt-1 to 25(OH)D ratio (with a similar cutoff value as above, 653) turned out to be a significant predictor of PE (*p* < 0.0001), with an AUC equal 87.96%. Based on these findings, it can be speculated that sFlt-1 and 25(OH)D not only play an important role in the pathogenesis of GH and PE but can also be used as predictors thereof. A similar character of relationships between sFlt-1 and 25(OH)D levels and the risk of GH and PE might be explained by the fact that both those factors interfere with vascular endothelium [30]. However, in our present study, 25(OH)D did not turn out to be an independent predictor of either hypertension or preeclampsia on multivariate logistic regression analysis (*p* > 0.05).

The authors of one previous study, Ma et al. [31], verified whether vitamin D supplementation alleviated PE-associated endothelial dysfunction and explored the underlying mechanism of this relationship using a reduced uterine perfusion pressure (RUPP) rat model. 1,25(OH)2D turned out to significantly downregulate the expression of placental sFlt-1 in RUPP rats. Furthermore, circulating sFlt-1 levels in maternal serum correlated positively with the expression of placental sFlt-1 and returned to normal values after supplementation with vitamin D. Based on those findings, the authors concluded that vitamin D supplementation might have protected against the RUPP-induced endothelial dysfunction by downregulating placental sFlt-1, which could plausibly alleviate PE-related symptoms.

Another study, conducted by Song et al. [32], verified whether vitamin D supplementation could restore angiogenic balance and ameliorate inflammation in a rat model for PE. Animals from the supplemented group presented with significantly higher concentrations of VEGF and significantly lower sFlt-1 and TNF-*α* levels than untreated rats with PE. Therefore, the authors concluded that vitamin D supplementation might play an important role in the restoration of angiogenic balance and attenuation of inflammation in pregnancy-induced hypertension [32].

Schulz et al. [33] demonstrated that sFlt-1 and VEGF gene expressions in the maternal subgroup with circulating 25(OH)D ≥ 100 ng/ml were significantly downregulated compared to the subgroup with 25(OH)D < 100 ng/ml. Moreover, they found a significant association between the maternal vitamin D status and the expressions of sFlt-1 and VEGF at the mRNA level. Based on those findings, the authors stated that maternal supplementation with vitamin D3 may exert an effect on gene transcription in the placenta and, thus, may reduce the level of antiangiogenic factors that are implicated in vascular pregnancy complications [33].

Only few previous studies analyzed sFlt-1 levels in women with GDM, and their results are inconclusive. In our present study, we found no differences in sFlt-1 levels in the GDM G1 and GDM G2 groups and the controls (4301 pg/ml vs. 3704 pg/ml vs. 3532 pg/ml, *p* = 1.00). One potential explanation for this phenomenon might be the fact that our patients with GDM still did not develop an endothelial damage, and thus, their sFlt-1 concentrations remained within the normal range. In our opinion, no ultimate conclusions can be formulated on the role of sFlt in GDM and this issue needs to be addressed in further studies [34].

In conclusion, this study showed that determination of the sFlt-1 to 25(OH)D ratio may facilitate the identification of patients with preeclampsia and gestational hypertension and their qualification for intensive treatment, which can be reflected by better neonatal outcomes.

The results of our study, which can be considered preliminary findings, justify further clinical research on a larger group of patients, including measurements of vitamin D concentrations to calculate the ratio derived from this parameter aside from that based on sFLT-1 and PLGF levels.

## Figures and Tables

**Figure 1:** ROC curve—relationship between sFlt-1 concentrations (pg/ml) and occurrence of gestational hypertension (AUC 70.1%).

**Figure 2:** ROC curve—relationship between sFlt-1 concentrations (pg/ml) and occurrence of preeclampsia (AUC 82.4%).

**Figure 3:** ROC curve—relationship between sFlt-1/25(OH)D index and occurrence of gestational hypertension (AUC 73.6%).

**Figure 4:** ROC curve—relationship between sFlt-1/25(OH)D index and occurrence of preeclampsia (AUC 87.96%).

**Table 1:** Baseline characteristics of the study participants.

Parameter	Study group (*N* = 171)	Control group (*N* = 36)	*p*
Age (years)	29.6 ± 5.2	29.4 ± 4.9	NS
BMI (kg/m^2^)	27, 8 ± 2, 2	26, 9 ± 2, 4	NS
Parity	1.9 ± 1.1	1.8 ± 1.0	NS
pH of umbilical artery	7.35 ± 0, 09	7, 35 ± 0.07	NS
BMI (kg/m^2^)	24, 8 ± 2, 0	25, 2 ± 2, 5	NS
Pregnancy (weeks)	38 ± 2, 96	40 ± 1, 08	NS
Caesarian sections (%)	43,3%	37,6%	NS
Weight of newborn (g)	3340 ± 680	3590 ± 430	NS
Systolic blood pressure (mmHg)	126,8 ± 13, 5	120,2 ± 9, 1	NS
Diastolic blood pressure (mmHg)	80, 3 ± 10, 3	76, 9 ± 8, 6	NS
GH status	*N* = 45	*N* = 0	—
Preeclampsia status	*N* = 23	*N* = 0	—
GDM status	*N* = 103	*N* = 0	—

**Table 2:** sFlt-1 concentration (pg/ml) in the group of patients with hypertension and the control group.

sFlt-1 (pg/ml)	Gestational hypertension (*N* = 45)	Control group (*N* = 36)	*p* value
Median range	5797 (4746-10277)	3531 (2672-4980)	*p* = 0.0014

**Table 3:** sFlt-1 concentration (pg/ml) in the group of women with preeclampsia and the control group.

sFlt-1 (pg/ml)	Preeclampsia (*N* = 23)	Control group (*N* = 36)	*p* value
Median range	6074 (5273-12448)	3531 (2672-4980)	*p* < 0.0001

**Table 4:** sFlt-1 concentration (pg/ml) in the group of patients with gestational diabetes and the control group.

sFlt-1 (pg/ml)	GDM G1 (*N* = 19)	GDM G2 (*N* = 84)	Control group (*N* = 36)	*p* value
Median range	4301 (2384-5977)	3704 (2403-5153)	3531 (2673-4980)	*p* = 1.0000

**Table 5:** sFlt-1 concentration (pg/ml) in relation to blood pressure.

	sFlt-1 (pg/ml)			
	RR > 140/90	RR > 160/100	RR > 180/110	Control group
Median	5399	5880	6074	3531
Range	(4048–8232)	(4443–9239)	(5176–12325)	(2672–4980)
*p* value (vs. the control group)	0.0055	0.0015	0.0059	

**Table 6:** sFLT-1 levels in the group of patients with sufficient serum concentrations of 25(OH)D (>20 ng/ml) and with vitamin D insufficiency/deficiency (25(OH)D ≤ 20 ng/ml).

	sFlt-1 (pg/ml)	
	25(OH)D (ng/ml) ≤ 20	25(OH)D (ng/ml) > 20
Median	4452	3356
Range	(3137.5–6066.75)	(2447–5284)
*p* value	0.0256	

**Table 7:** Relationships between serum concentrations of sFlt-1 and the incidence of gestational hypertension (GH) and preeclampsia (PE); results of ROC (receiver operating characteristic) analysis.

Parameter	GH	PE
AUC	0.7012	0.8237
SE (AUC)	0.0489	0.0488
-95% CI	0.6055	0.7280
+95% CI	0.7970	0.9194
*Z*-statistic	3.9942	4.9837
*p*	0.0001	<0.0001
Cutoff value	9643	10488

**Table 8:** Relationship between serum concentrations of sFlt-1/25(OH)D index and the incidence of gestational hypertension (GH) and preeclampsia (PE); results of ROC analysis.

Parameter	GH	PE
AUC	0.7359	0.8796
SE (AUC)	0.0483	0.0354
-95% CI	0.6413	0.8101
+95% CI	0.8306	0.9490
*Z*-statistic	4.5472	5.6978
*p*	<0.0001	<0.0001
Cutoff value	652.37	653.19

**Table 9:** Results of multivariate logistic regression analyses examining the effects of serum sFlt-1 levels (pg/ml), BMI ≥ 30, age ≥ 35, primiparity, and 25(OH)D ≤ 20 ng/ml on the incidence of hypertension.

Parameter	*b*-coefficient	*p* value	Odds ratio	-95% CI	+95% CI
Intercept	-2.7821	0.0071	0.0619	0.0082	0.4687
sFlt-1 (pg/ml)	0.0004	0.0170	1.0004	1.0001	1.0007
BMI ≥ 30	2.7985	0.0003	16.4199	3.5615	75.7012
Age ≥ 35 years	-0.5656	0.5221	0.5680	0.1005	3.2093
Primiparity	0.6656	0.3842	1.9456	0.4345	8.7132
25(OH)D ≤ 20 ng/ml	0.1091	0.8875	1.1153	0.2459	5.0592

**Table 10:** Results of multivariate logistic regression analyses examining the effects of serum sFlt-1 levels (pg/ml), BMI ≥ 30, age ≥ 35, primiparity, and 25(OH)D ≤ 20 ng/ml on the incidence of preeclampsia.

Parameter	*b*-coefficient	*p* value	Odds ratio	-95% CI	+95% CI
Intercept	-5.6590	<0.0001	0.0035	0.0005	0.0250
sFlt-1 (pg/ml)	0.0004	0.0001	1.0004	1.0002	1.0006
BMI ≥ 30	0.6718	0.2829	1.9578	0.5745	6.6724
Age ≥ 35 years	-1.5500	0.2223	0.2122	0.0176	2.5585
Primiparity	0.9548	0.1540	2.5982	0.6991	9.6559
25(OH)D ≤ 20 ng/ml	1.0028	0.1331	2.7259	0.7365	10.0883

## Data Availability

The data used to support the findings of this study are available from the corresponding author upon request.
